The article "“Recovering With Nature”: A Review of Ecotherapy and Implications for the COVID-19 Pandemic" was retracted in 2023. Reason: compromised peer review.

# “Recovering With Nature”: A Review of Ecotherapy and Implications for the COVID-19 Pandemic

**DOI:** 10.3389/fpubh.2020.604440

**Published:** 2020-12-10

**Authors:** Pourabi Chaudhury, Debanjan Banerjee

**Affiliations:** ^1^Department of Clinical Psychology, Institute of Psychiatry (IOP), Kolkata, India; ^2^Department of Psychiatry, National Institute of Mental Health and Neurosciences (NIMHANS), Bengaluru, India

**Keywords:** ecosystem, ecotherapy, psychology, mental health, nature, COVID-19

## Abstract

Connection with nature has been considered beneficial for psychological well-being since times of evolution. Differences in Indian and Western thoughts have viewed natural elements in different lights, varying between eco-centrism to anthropocentrism. The intrusion of technology and digitalized lives as a result of globalization has decreased connectedness with nature. Ecotherapy is a novel form of psychotherapeutic technique based on explicit environmental or ecological interventions. Social and therapeutic horticulture, animal-assisted interventions, care farming, green exercise, environmental conservation and wilderness therapy are some of the ecosystem-based approaches used in mental health. Based on the principles of positive and client-centered psychology, ecotherapy-related techniques have been shown to be effective in medical disorders like hypertension, obesity, post-surgical recovery and psychosocial conditions like depression, stress reduction, post-traumatic stress disorder (PTSD), attention deficit hyperkinetic disorder (ADHD) and adjustment disorders. The principles of ecotherapy have been integrated into other psychotherapeutic techniques for better efficacy. This review attempts provides an overview of techniques, applications and challenges related to ecotherapy in psychology. The implications of its use during the ongoing Coronavirus 2019 (COVID-19) crisis, social isolation and consequent psychosocial aftermath are also discussed.

## Introduction

The conception that man is an integral and indispensable part of nature with mutually nourishing existence has been emphasized in Indian philosophy since time immemorial. Indian thought has always given prominence over the fact that man and nature are not radically different entities. Hence in ancient Indian tradition there was restraint in utilization of natural resources to desirable needs and necessities. Nature was not perceived as a commodity to be consumed for human fulfillment. Nature was worshiped and considered sacred and there has been reasonable harmony between man and nature (1). Certain Western thoughts desacralized nature and conceived environment as a utilitarian agency. Permission was given to exploit natural resources with no regard for consequences. Man and nature were considered as different entities with man having the supreme power to interfere in the natural discourse of nature. With the intrusion of colonial power the concept of human-centered philosophy gripped the Indian society as well. Gradually eco-centrism was replaced by anthropocentrism (1, 2). Globalization, urbanization and technological advancements retreated man further from the “Great outdoors” to the gadget oriented world of televisions, computers and gaming; and accelerated the pace of ecological disequilibrium on an unprecedented scale (3, 4). This shift led to a decrease in exposure to natural environments (5, 6). There is also evidence of an increase in the worldwide prevalence of mental disorders concurrent with urbanization (7, 8). These two trends may be linked with decreased exposure to nature causing changes in psychological functioning as suggested by growing evidence (9, 10). Thus, along with rapid depletion of our natural resources beyond limits that can be replenished, our psychological framework has also been affected which has already been neglected long enough. Research in the recent past has been consistently showing how contact with nature enhances various aspects of well-being (11–14). However, for most it took a pandemic and the consequent home confinement to be not only reminded of mankind's barbaric and unpardonable acts of destroying ecological balance and it's interdependent relationship with mankind but also for the realization to set in that how interaction with nature can soothe us, create positive affect, elevating experiences and a general sense of connectedness to life as a whole (15). During this COVID-19 pandemic when man is restricted within the periphery of his residence and nature has started reclaiming itself through reappearance of species that were rarely to be seen, many of us are discovering new birds, observing the crimson rays of the setting sun, being enthralled by the freshness of the morning air when the first ray of a new day welcomes us with hope for a brighter future or may be nurturing our houseplants, all of which are making us feel better. Keeping this in background, this review attempts to address the following questions: How can we adopt an ecological approach toward psychosocial well-being? How can such “active involvement with nature” be structured into mental health interventions? How can these therapeutic interventions focused on “reconnecting back with nature” be beneficial in improving emotional health during the COVID-19 crisis?

The article "“Recovering With Nature”: A Review of Ecotherapy and Implications for the COVID-19 Pandemic" was retracted in 2023. Reason: compromised peer review.

## COVID-19: Global Problem Statement

The adversity following COVID-19 pandemic that billions around the globe is going through was inevitable and much foreseen after its outbreak was declared as a Public Health Emergency of International Concern (PHEIC) by the World Health Organization on January 30, 2020 (16). The global count of confirmed cases of COVID-19 is nearing 19 million with more than seven lakh deaths worldwide, according to the World's Health Organisation's latest report (17), with numbers steeply rising as each day passes. The scenario in India being no less alarming shows that the number of confirmed cases has crossed the 21 lakh mark with over 43,000 deceased individuals (18). An outbreak with such extensive repercussions will unquestionably have its influences on mental health and wellbeing besides the physical health parameters (19, 20).

## COVID-19, Social Distancing and Psychological Well-Being

Originating in the Wuhan City of the Hunan Province of China in month of December, 2019, this Coronavirus disease (COVID-19) has been spreading like wildfire (16) and taking a toll on the lives of every individual across the globe irrelevant of the socioeconomic strata. In order to restrain the propensity of spread of SARS-Cov-2 the entire world has adopted various containment measures starting from quarantine, social distancing, self-isolation and travel restriction. Since early February, 2020 travel ban has been implemented in Wuhan City and international travel restrictions have been adopted by several countries (21). In March, 2020, the Government of India also took the decision of a historical National Lockdown in order to curb community transmission in which traveling to various parts of the country by any individual was entirely put to a halt. That all these restrictive measures following the pandemic have affected not only physical health but also have posed a detrimental impact on mental health and well-being, has been widely talked about and accepted (19, 20). It is a known fact that reduced social interactions and increased loneliness are well-known risk factors for several mental disorders, including major depression, anxiety, post-traumatic stress and schizophrenia. Apprehension regarding one's own health and that of their beloved ones (particularly elderly or individuals suffering from any physical illness), as well as immense unpredictability related to future circumstances, can exacerbate fear, depression, and anxiety. Prolonged exposure to these concerns, may increase the risk of serious and disabling mental health conditions including anxiety disorders like panic, obsessive–compulsive, stress, and trauma-related disorders (22). Again after studying emotional indicators (e.g., anxiety, depression, indignation, and happiness) and cognitive indicators (e.g., social risk judgment and life satisfaction) before and after the declaration of COVID-19 on January 20, 2020, the same group of researchers reported that negative emotions (e.g., anxiety, depression and indignation) and sensitivity to social risks increased, while the scores of positive emotions (e.g., happiness) and life satisfaction decreased (23). Researches also indicated high prevalence of mental health problems (depression, anxiety, and combination of depression and anxiety), which were positively associated with frequent social media exposure during this COVID-19 outbreak (24). Hence, measures to mitigate these mental health consequences demands utmost priority before the aftermath of this pandemic gets even worse.

The article "“Recovering With Nature”: A Review of Ecotherapy and Implications for the COVID-19 Pandemic" was retracted in 2023. Reason: compromised peer review.

## Infectious Disease Outbreaks and Ecological Balance: the Intersections

The prevalence of human diseases has changed in type as humans shifted from hunting-gathering, to agriculture finally to urbanization during Industrial Revolution. Research indicates that globalization and ecological disruption have culminated in the recent emergence and re-emergence of infectious diseases. Researchers opined that increase in the incidence and distribution of infectious diseases affecting humans may have resulted from habitat destruction and biodiversity loss associated with biotic homogenization. The spread of non-indigenous vectors and pathogens establishes a clear connection between biotic homogenization and infectious disease. Further the increase in incidence of vector borne illnesses may be attributed to the loss of predators and hosts that dilute pathogen transmission. Enhanced abiotic conditions for pathogens and vectors and higher host-pathogen encounter rates are among the other mechanisms that accelerate the incidence of infectious diseases (25) Again biotic homogenization can result from anthropomorphic pressures like urbanization which can also have profound impacts on biota, leading to changes in assemblages (26). Further natural selection and other evolutionary forces that lead to extinction can also potentially lead to homogenization (27). There have been various takes on the ecological balance, impact of climate and their intersections with infectious disease outbreaks. The recent-most example is that of COVID-19 and the consequent lockdown that has affected air-emissions, pollution, water quality, plastic use, environmental quality and socio-ecological balance (28). Animal and plant lives have been rejuvenated and were more visible during the global lockdown. This does not imply that an infection is necessary for the ecological balance, but rather that our consistent tampering with the systems of nature have led to the evolutionary basis of pathogens and maintenance of infectious outbreaks. There has been evidence that wildlife trafficking may have played a role in the first emergence of the ongoing pandemic in a wet market in Wuhan, China which has now claimed more than a million lives globally (29). Similar illnesses like the Severe Acute Respiratory Syndrome (SARS) and the Middle East Respiratory Syndrome (MERS) have had associations with sales of wild animals and climate alterations (30). An important concern during the 2009 H1N1 influenza was the massive factory farm industry, which could have possibly influenced the efficacy of antibacterial medications or have led to pathogen-mutations (30). Restoring the ecosystems has been mentioned in many strategies for dealing with the COVID-19 and also the post-pandemic aftermath. Zabaniotou (31) while discussing the uncertainty and stress of the COVID-19 pandemic, emphasizes on the importance of preserving bio-diversity, enhancing bio-capacity and conceptualizes various frameworks of resilience by promoting a holistic health of the planet. The positive insights gained from the pandemic are viewed through the transdisciplinary lens of social and ecological solidarity that can facilitate a resilient globalization, coping and help mitigate the growing uncertainty. Balancing the planetary health and bio-capacity along with human economy and consumerism is thus vital for fighting a global biological crisis like COVID-19. Lessons learnt during this outbreak by viewing the bio-psychosocial distress from an ecological point of view can serve as a preparedness tool for futuristic crisis. Banerjee and Nair (32) while proposing a community-based toolkit for the ongoing pandemic based on the earlier World Health Organization (WHO) model for the Zika virus outbreak stressed on the importance of community involvement in preservation of environment, climate and wildlife as an integral part of public health to deal with the crisis situations besides just a medical or psychological approach. Based on the Intergovernmental Science-Policy Platform on Biodiversity and Ecosystem Service (IPBES) Global Assessment Report 2019, more than 75% of the terrestrial environment has already been impacted by urbanization. Since deforestation and biodiversity loss are considered to be facilitators of zoonoses (diseases transmitted from animals to humans), long-term ecological solutions including nature-conservation, prevention of deforestation, ban on wildlife trade and live animal markets need to be a part of public-health surveillance, strategies and policies (30). In this paper, we predominantly discuss the ecological approach to psychological well-being and its implications during the ongoing pandemic. Adequate understanding of the gap with our wider world and the vicious acts of human beings is a priority for protecting human health wherein the emerging field of ecotherapy may have potential usefulness.

The article "“Recovering With Nature”: A Review of Ecotherapy and Implications for the COVID-19 Pandemic" was retracted in 2023. Reason: compromised peer review.

## Ecotherapy as a Novel Approach in Psychology

It is often experienced that a simple walk in a park, observing a plant sprouting to life from a tiny seed or going on vacation far away from the hustle of the city has at least partially relieved people the from overwhelming stress that we might be into and made people feel new again (33). This gives us a clear indication that man indeed has a deep rooted desire to connect back to the natural world however much he separates himself from it, in his technologically advanced, sophisticated, well-furnished residence. In Erich Fromm's words “I believe that man is the product of natural evolution that is born from the conflict of being a prisoner and separated from nature, and from the need to find unity and harmony with it” (34).

### A Look Into the Evolution of Ecopsychology and Ecotherapy

“*Psychology, so dedicated to awakening human consciousness, needs to wake itself up to one of the most ancient human truths: we cannot be studied or cured apart from the planet.”*

James Hillman (35)

The human-to-nature relationship has been mostly omitted in psychology literature. According to clinical psychologist Ralph Metzner this omission has been addressed by the new field of “ecopsychology (36). This nascent field of ecopsychology is a bairn of the environmental movement which began in the 1960s in response to the dawning recognition that modern industrial civilization had engendered an environmental crisis. Though it is difficult to demarcate the time and distinct person responsible for the emergence of ecopsychology, certain formative events and persons are particularly noteworthy.

The origins of ecopsychology can be traced to Robert Greenway, who coined the term “psychoecology” in 1963 (37). Paul Shepard, has also been credited with pioneering the study of ecopsychology with the publication of his “Nature and Madness” in 1982 (38). Inspired by Greenway's teachings Theodore Roszak in 1992, coined the term ecopsychology that was outlined in his “Voice of the Earth,” which he considers an essay in ecopsychology (39). Ralph Metzner is also considered one of the founders, ostensibly because of his many eco psychological essays, and his early courses in the subject (40). Harold Searles is considered by some to be “a proto-eco psychologist” for postulating the importance of ecologically healthy relatedness to our non-human environment and encouraging psychoanalysts to make contribution toward meeting the ecological crisis (41).

The article "“Recovering With Nature”: A Review of Ecotherapy and Implications for the COVID-19 Pandemic" was retracted in 2023. Reason: compromised peer review.

Roszak has postulated a broad definition of ecopsychology: (1) Ecopsychology is the emerging synthesis of ecology and psychology. (2) It is the skilful application of ecological insights to the practice of psychotherapy. (3) It further encompasses the discovery of our emotional bond with the planet. (4) It defiens “sanity” as if the whole world mattered. According to his opinion as a psychology it seeks to comprehend humankind's interrelationship with the non-human world, to diagnose what is wrong with that interrelationship, and to suggest paths to healing (35).

Roszak had a dual purpose of adding “eco” to “psychology” in 1992. The first purpose being that conventional psychology is in desperate need of re-conceptualizing its theory and practice within an ecological context if it intends to impact constructively the environmental crisis. The second purpose, was that the environmental movement is in dire need of “a new psychological sensitivity” and has much to learn from psychology about how to motivate people to change their environmentally destructive behavior. Various other researchers have subsequently defined ecopsychology which builds upon the basic premise put forward by Roszak (39).

The term ecotherapy was first coined by Clinebell (42) and he propounded it as a form of ecological spirituality, where a holistic relationship with nature embraces both nature's tendency to foster us through our contact with natural places and our ability to reciprocate this remedial connection through our ability to nurture nature. He attempts to differentiate his notion of ecotherapy from ecopsychology: “Ecotherapy refers to both the healing and the growth that is nurtured by healthy interaction with the earth,” whereas ecopsychology refers “to what is called the ‘greening of psychology”' (42). Roszak however, incorporates ecotherapy in ecopsychology; that is, he intends “to embrace the psychotherapeutic and the psychiatric” (43).

### Basic Principles of Ecopsychology

In “The Voice of the Earth,” Roszak put forth a list of principles for ecopsychology:

- The ecological unconscious is in the core of our mind and the repression of which is collusive madness and open access to it is the path to sanity.
- The ecological unconscious consists of the living record of cosmic evolution.
- The ecological unconscious contains an inherent sense of environmental reciprocity which when awakened can heal the alienation between person and environment.
- Ecopsychology attempts to unravel the child's intrinsic animistic quality of experience in functionally “sane” adults” and to create the “ecological ego.
- The ecological ego matures to develop a sense of ethical responsibility with the planet.
- We need to re-evaluate certain compulsively “masculine” character traits that drive us to dominate nature.
- Ecopsychology is post-industrial not anti-industrial in its social orientation.
- The needs of the planet are the needs of the person, the rights of the person are the rights of the planet (39).

The article "“Recovering With Nature”: A Review of Ecotherapy and Implications for the COVID-19 Pandemic" was retracted in 2023. Reason: compromised peer review.

### Elucidating Ecotherapy in a Nutshell

Thus in the last decade of the twentieth century the connection between man and nature coalesced as a discrete endeavor in the form of explicit environmental or ecological initiatives in counseling and psychotherapy termed “Ecotherapy” (44–46). The Mind evaluation report on Ecotherapy (sometimes called GREEN CARE) drafted by the University of Essex states that “Ecotherapy comprises nature based interventions in a variety of natural setting” (2). Thus, it is one of the ecosystem services that nature provides and refers to the treatment modalities that include the natural world in relation to mutual healing and growth, and as such is a form of applied ecopsychology. Broadly speaking it is an area of social psychiatry and psychology that embrace social determinants of mental health, psychology and ecology with the aim to be holistic in theory and practice (47). From an ecotherapy perspective this means that, the bio-psychosocial health of a human being is viewed in the context of the health of the Earth and its natural ecosystems (42). Ecotherapy helps people connect with nature to assist in dealing with physical and mental illnesses (48). This idea of reconnection seeks to evoke in humans that we are an integral part of ecosystems rather than separate from them (49, 50). Although flowering of ecotherapy initiatives originated in the western world it brings back the age old Indian philosophy of inseparable existence of man and nature.

There has been ambiguities around the term “ecotherapy” (51) and the term “green care” has been proposed to be used as an overarching word for all types of therapeutic activity related to nature, animal, and plants (52). Although ecotherapy is a more commonly used term and its generic use applies to any facilitated activity that is related to nature (plants, animals, and landscape) and as such will encompass many activities in nature such as conservation work, mountaineering and rambling that indeed has positive effects, however specifically it refers to interaction with wild and natural areas of nature and enhancing the positive effect of natural surrounding on affect and cognition through increasing sensory contact and mindfulness (2). Although confusion still exist regarding what the broader terminology would be, The Natural England Review of nature based interventions for mental health care (53) adopts “green care” as the umbrella term that embraces various subgroup. For ease of understanding, we will adhere to the term ecotherapy in the general sense as a broader terminology in our further discussions in this article.

The article "“Recovering With Nature”: A Review of Ecotherapy and Implications for the COVID-19 Pandemic" was retracted in 2023. Reason: compromised peer review.

Some of the main subgroups following McGeeney (2) are summarized in Table 1.

**Table 1:** Various subtypes of ecotherapy / “green care”: applications, evidence and utility during COVID-19.

**Types**	**Attributes**	**Applications and evidence**	**Potential utility during the COVID-19 pandemic**
Social and therapeutic horticulture	It is the most popular therapeutic interaction between people and plants. It can be passive appreciation of a garden, active gardening or growing vegetables	• Improving mood state (54); fostering emotional restoration (55) • Reduction of stress (54, 56) • Modifying progression of coronary heart disease by addressing associated anxiety and stress (54) • Improving self-esteem and reduce depression (57, 58) • Improving sleep and cognitive issues in dementia patients (59) • Increasing engagement and improving mood-related to dementia (60, 61) • Treatment of substance abuse (62) • Restoration of attention in cancer patients (63) • Dealing with service-provider burnout (64) • Reducing isolation felt by the elderly (65)	• Dealing with the stress, anxiety, loneliness and uncertainty of the pandemic • For people living alone, in isolation, quarantined and significant restriction of movement Especially for older adults and children (who need more social and cognitive stimulation) • Dealing with grief, adjustment disorders, depression, anxiety disorders
Animal-assisted interventions	This includes activities with pets, horses and other domesticated animals Animals have been used for a variety of therapeutic interventions to improve well-being and self-esteem. An important aspect of this intervention is that a pet animal such as a dog is likely to be friendly and affectionate to anyone and it does not approach human being with any prejudices	• Improving vitality, emotional balance, extraversion, and alertness in children and adolescence (66) • Decreasing aggressive behavior in children (67) • Decreasing aggression and agitation in elderly (48) • Reducing physiological stress in children (68) • Decreasing anxiety, lower physiological arousal, increased social interaction for survivors of sexual abuse suffering from posttraumatic stress (69) • Decreasing agitation and aggression in Alzheimer's patients (70) • Decreasing loneliness (71), reducing depressive symptoms (72) • Preventive medicine against the risk of cardiovascular disease (73) • Useful in schizophrenia, anxiety, affective disorders, and personality disorders in improving in coping ability, self-efficacy, symptom reduction, and quality of life (74)	• Effective to deal with stress, anxiety originating from uncertainty of the current situation, • Calming aggressive feelings, decreasing loneliness • Bringing alertness and emotional balance in children in this ongoing situation of COVID-19
Care farming	This is the therapeutic use of agricultural landscapes and farming practices (51). It covers a variety of contexts and farm related activities such as looking after animals, vegetable growing and crop management	• Improving self-esteem and mood (75–77) • Rehabilitation for alcohol or drug addiction (76, 77) • Improving well-being, increase in self-confidence and calmness (76, 77)	• Not applicable in the current context
Environmental conservation	This includes engaging in conservation work for the improvement of health and well-being	• Improving mental and physical health (78, 79)	• Not applicable in the current context
Green exercise	Along with walking and other physical exercise outdoor in parks and the countryside, the focus here is also on socializing like appreciating the natural world (80)	• Improving personal well-being, mental and for physical health benefits (81, 82) • Decreasing anxiety, rumination, negative affect, and preservation of positive affect (83) • Cognitive benefits like increased working memory performance (83)	• Physical activity and outdoor engagement with nature-rich environments in the local proximity of residences (parks and gardens are ideal; again needs to be practiced with the necessary social distancing) are beneficial for enhancing well-being and reducing stress during this calamity.
Nature arts and crafts	This is drawing, painting, photography writing poetry etc. outdoors in parks or countryside	• Improving mental health and wellbeing (2)	• Writing, painting, photography, planting, designing and crafts (with the usual precautionary measures of COVID-19) fosters positive mental health.
Wilderness therapy	Interaction with nature by an individual or group in remote location leading to self-discovery and change	• Useful in PTSD treatment (84) • Reducing stress (85) • Adolescent behavior problem (86) • Promoting self-esteem, behavior change, and interpersonal skills in juvenile delinquents (87) • Increasing self-esteem in children (88) • Substance abuse treatment (89) • Treating self-esteem issues, schizophrenia, mood modification, anger management, (90) • Family functionality and well-being (91, 92)	• Not applicable in the current context
Specific ecotherapy techniques	The central assumption here is that nature itself is the primary therapeutic source. Here interaction occurs with wild or semi-natural areas of nature. The process is enhanced through sensory contact and mindfulness	• Accelerating medical recovery rates after surgery (93–96) • Useful in healthcare facility design targeted to reduce pain (97) • Useful in PTSD treatment [(98), Dustin et al., 2011] • Used in mood modification and stress reduction (99) • Widely effective in reducing attention deficit symptoms in children (100, 101) • Psychosocial management in dementia (102); decreasing agitation in dementia (103) • Improving individual's well-being (104, 105)	• Interactions with bird, wildlife, plants (in various forms), social connectedness, experiencing nature and cherishing the memories of such interactions (like photography, videos, etc.) helps in dealing with loneliness and strengthens well-being.

The article "“Recovering With Nature”: A Review of Ecotherapy and Implications for the COVID-19 Pandemic" was retracted in 2023. Reason: compromised peer review.

## Theoretical Models of Ecotherapy

To explain how our relationship with nature plays a fundamentally important role in our well-being several theoretical models and perspectives have evolved. The “Biophilia Hypothesis” (106–108) suggests that human identity and personal fulfillment depend on our relationship with nature. Comparable to the meaning of the word biophilia (love of life), the hypothesis contends the existence of a fundamental, genetically based human need and inclination to affiliate with and respond with emotional intensity to non-human natural world. Fromm (109) believed that a productive, creative, caring attitude toward life is fundamental to our own mental health and for humankind as a whole, if it has to survive. He opined that biophilia is the essence of humanitarian ethics. According to Wilson (108), the biophilic instinct emerges, in our cognition, emotions, art, and ethics, often unconsciously, and unfolds “in the predictable fantasies and responses of individuals from early childhood onward. It cascades into repetitive patterns of culture across most or all societies.”

The Eco-Existential Positive Psychology perspective, expanding on this hypothesis, (110) proposes that cultivating our innate biophilic tendencies through involvement with the natural world enhances our well-being by helping us manage our existential anxieties, such as those concerning isolation and happiness.

Attention Restoration Theory (ART) suggests that, urban environments profusely rests upon the top-down voluntary attentional control that is required to filter relevant from irrelevant stimuli adequately. Thus, cognitive resource are depleted from demands from the urban environment, and can thereby worsen, directed performance on tasks that rely on this focused attention (111, 112). According to ART, natural environments elicit a different sort of attention from people—a sense of “fascination,” and “being away,” and “compatibility”—the outcome of which is the replenishment of directed attention because natural environments are rich in stimuli that effortlessly engage our involuntary attention (“soft fascination”) and thus restore our directed attention/cognitive capabilities (112, 113). In turn, this may lead to improved performance on tests that measure memory and attention.

The article "“Recovering With Nature”: A Review of Ecotherapy and Implications for the COVID-19 Pandemic" was retracted in 2023. Reason: compromised peer review.

Stress reduction theory (SRT) provides a clarification for the impact of nature experience on affect. This theory proposes that natural environments have a restorative advantage over artificial environments due to the role that they played in our evolution as a species (114). According to this view, nature scenes activate our parasympathetic nervous system and in turn reduce stress and autonomic arousal. This calming effect is brought about because of our innate connection to the natural world. According to Ulrich et al. (93, 94), viewing natural landscapes (especially grasslands with clusters of trees) in particular activates our physiology in affectively beneficial ways, as we have evolved to have an innate preference for these types of environments. Hence a set of testable hypotheses regarding nature's impact on the autonomic nervous system is provided by Ulrich's theory, and these have been tested via the use of physiological measurements of individuals during their exposure to various environments. In order to test these hypotheses, R.S. Ulrich examined the psychological influence of stress experienced by students on being exposed to scenes of nature (107, 114–116) and medical recovery rates (117). Findings revealed increased positive feelings of friendliness, affection, joy and playfulness when they observed “natural” scenes. Viewing urban scenes resulted in primarily feeling of sadness along with a tendency to increase feelings of anger. When brain activity in healthy, unstressed adults was measured it demonstrated that viewing landscapes that were associated with nature resulted in the increased production of serotonin, the “happiness-promoting” neurotransmitter (93, 94). Many antidepressant medications are thought to work by elevating the availability of serotonin in the limbic system and pre-frontal cortical circuitry. Objective testing to confirm this phenomenon have been conducted by many subsequent researches. Ulrich's landmark research showed changes in surgical recovery time based on patients' window views of nature (trees) and urban scenes (walls, concrete) demonstrating that this “natural” capacity extended beyond feelings to detectable medical phenomena (33).

The article "“Recovering With Nature”: A Review of Ecotherapy and Implications for the COVID-19 Pandemic" was retracted in 2023. Reason: compromised peer review.

Table 2 summarizes a look into the role of ecosystem services in therapies for several disorders and overall developmental approaches.

**Table 2:** Research evidence for Ecotherapy in various disorders.

**Physical and mental health disorders**	**Research evidence**
Medical Recovery	✓ Enhanced recovery rates of patients undergoing appendectomies were attributed to flowering plants and foliage in hospital rooms (95) ✓ Generalized enhanced health outcomes in patients recovering from surgery were linked to indoor ornamental plants (96) ✓ Enhanced mental health recovery rates of coronary and pulmonary patients were associated with indoor plant exposure in Norway (118)
Pain Reduction	✓ Bio monitoring experimental sessions revealed increases in pain tolerance as a result of exposure to ornamental plants in a simulated hospital room (119) ✓ In a randomized clinical trial of patients undergoing flexible bronchoscopies combining nature sounds and images was shown to reduce pain (120) ✓ Exposure of increased levels of sunlight for patients having undergone spinal surgery resulted in reduced pain, stress, and use of painkilling medication (121)
Post-traumatic Stress Disorder (PTSD)	✓ Wilderness therapy, outdoor adventure and experience and green-space based ecotherapy (e.g., river rafting, interactions and participation in nature) have been shown to be effective therapeutic media for veterans coping with PTSD (84, 122)
Mood Modification, Stress Reduction	✓ Horticultural therapy has been shown to improve mood state reducing stress and positively contribute to coronary heart disease (54), improve self-esteem and reduce depression (57, 123). Healing gardens and natural ecosystem encounters have been shown to reduce depression (58), reduce stress (124) ✓ Spending time in nature, green exercise show positive effect on people's self-esteem and mood (82, 125)
Substance Abuse	✓ Horticultural activities (62) and integrated adventure therapy programs (89), have been shown to be useful in substance abuse treatment ✓ Wilderness and outdoor experiences has been quite useful with chemical dependency (126)
Attention Deficit Hyperkinetic Disorder (ADHD)	✓ Improvement in motor ability, concentration and social play are all positively influenced following interaction or play in nature in children with ADHD (101) ✓ Increased green outdoors activities result in reduced children's ADHD symptoms and have more positive affect effects on symptoms than activities in other settings (100) ✓ Adults and children tend to perform systematically better on objective attention measures after viewing or spending time in natural surroundings (101)
Dementia	✓ The modification of dementia residential design plans in order to incorporate plants, nature and gardens have shown positive effects (127) ✓ Environmental psychologists have shown that exposure to nature and natural settings decreases agitation (61, 103) which often occurs in late stage of dementia ✓ Horticulture therapy improve sleep and cognitive issues in dementia patients (59), improve engagement and mood-related to dementia (60)
Obesity	✓ People with ready access to nature are less likely to be obese, inactive (128) ✓ Increased vegetation and green space were reported to be associated with reduced weight (129) ✓ In eight major European cities, people were 40% less likely to be obese in the greenest areas of those cities (130)
Overall development	✓ Direct contact with nature significantly and positively impacts children's affective, cognitive, and moral development (131, 132) ✓ The greener a child's view from their apartment, the higher he or she scored on several measures of delay of gratification and impulse control (133) ✓ Many studies suggested a systematic relationship between outdoor curricula in green space and enhanced learning (134, 135) ✓ Research into childhood outdoor experiences has identified that a key benefit of interaction with ecosystems is increased cognitive functioning (136, 137)
Well-being, life satisfaction	✓ Even short-term walking interventions, particularly in green-spaces, energize and enhance personal well-being and vitality (81, 138, 139) ✓ Research has established a strong link between contacts with nature and enhanced human well-being (105) ✓ One of the most useful applications of wilderness and outdoor experiences has been with the improvement of family functionality and well-being (92, 140) ✓ Interaction and engagement with green space have been linked with increased length of life and deceased risk of mental illness across a number of countries (99)

The article "“Recovering With Nature”: A Review of Ecotherapy and Implications for the COVID-19 Pandemic" was retracted in 2023. Reason: compromised peer review.

## Implications of Ecotherapy in COVID-19 Crisis

The upheaval caused by the COVID-19 pandemic and its repercussions on mental health have already been discussed. Though the concerns in the various vulnerable sections of the society may vary in its nature and intensity, some aspects may be comparable amongst all. For those who are quarantined, in home isolation or self-isolation and staying alone away from home, even passing a day might be distressing and traumatic owing to confinement, separation from loved ones, boredom, daily schedule getting haywire and feelings of loneliness. Added to that are the panic and fear of infection, the lockdown, financial crises and uncertainty. On the other hand for the elderly: apprehension regarding ailments one is suffering from, concerns regarding increased susceptibility to contamination and possibility of health deterioration, emergency service access and delivery of daily necessities might be a nerve-racking ordeal along with being perturbed about off springs living away and sometimes in high-risk areas. Loneliness which may be commonly experienced in this group in general may be further escalated due to restrictions imposed on gatherings and socialization in their own circle. Increased behavioral problems, attachment and emotional issues may become sources of worry in children for whom the two most significant activities—attending school and outdoor play have ceased to exist. The significance of the anxiety bothering every mind irrespective of any divisions cannot be over-emphasized.

It has been deliberated how over the past two decades a substantial body of research on nature-based intervention has developed which is gradually spreading its roots deeper through evidence-based approaches in establishing itself as an alternative mode of treatment in various physical and mental health concerns. In the light of its efficacy in dealing with depression, anxiety and stress, certain methods or techniques of this mode of intervention may be beneficial for dealing with the crisis that culminated from the present calamity are mentioned below.

### Possible Applications of Various Types of “Green Care”/Ecotherapy During COVID-19

- Social and therapeutic horticulture

This can be employed to deal with depressive feelings, loneliness in adults particularly the elderly stemmed from being quarantined or home confined. In increasing attentive capacity in children whose behaviors have been tremendously restricted. To tackle the stress and anxiety associated with this pandemic it can also be effective.

- Animal-assisted interventions

This can be extremely effective to deal with stress, anxiety originating from uncertainty of the current situation, calming aggressive feelings, decreasing loneliness and bringing alertness and emotional balance in children in this ongoing situation of COVID-19.

- Green exercise

It can be practiced individually by those people residing outside containment zones to improve overall well-being and reduce stress. Walking or other physical activity must be practiced in locations with hardly few people around and needed containment measures of COVID-19 should be followed.

- Nature arts and crafts

For facilitating better mental health during this crisis situation; writing, painting or photography outside can be practiced. However it must be done alone following containment measures of COVID-19.

- Specific ecotherapy techniques

Some of activities that can be employed in the ongoing COVID-19 situation to enhance psychological well-being and overcome loneliness are: listening to birdsong; bringing nature into your home through making bird-feeder, hanging nature picture and bringing home potted plants; experiencing nature by bringing back a strong memory of nature; getting to know another form of life by spending time with it and appreciating the good things in our lives at the moment.

The article "“Recovering With Nature”: A Review of Ecotherapy and Implications for the COVID-19 Pandemic" was retracted in 2023. Reason: compromised peer review.

The above-mentioned propositions do not form an exhaustive list and can be modified and tailored based on various environmental milieu and socio-cultural contexts.

According to Andy Fisher, mainstream mental health remains too entrenched in mind–body and self–world dualisms to explore the lived relationship between the human and the non-human, as is true for most environmental psychology practices (141). Much of the early writings reflects the presence of our alienation from the place we originally belonged to (142) and Chalquist (48) aptly refers it to a wall that divides self and others, person and place and thus self and Earth. Traditional psychotherapeutic approaches may develop more rationalities in thinking, foster new attitudes or habits still remaining confined to settings of urban alienation. However, through eco-therapeutic approaches a latent love for the world may be surfaced, we may be restored as a sensitive being with needs of its own and able enjoy a fulfilling healthy life through our homecoming, that is through reconnecting ourselves with rest of the Earth (48).

Talking specifically about various techniques stated above that may be beneficial during this time of need in fostering mental health and alleviating sources of distress, therapeutic horticulture may be the most fundamental and best-suited approach. For those who have a garden/space adjoining their houses regular tendering of their plants is a convenient option. For the rest modifying the balconies and window seal as a breeding ground for the greenery may bring in emotional satisfaction. Again, animal-assisted intervention is an appropriate alternative for the privileged families who already have a pet at home or a domesticated animal. They can encourage children and elderly to spend more time with the pets ensuring safety and may even plan out games and recreational activities. Drawing, painting, photography, as well as writing poetry are common media through which one can reconnect back with the wider world and experience a sense of belongingness. Sometimes natural materials like dried stems or leaves can be creatively employed in crafts and games (2). We must remember here that it's not about the quality of creativity but our sheer expressions, contexts and experiences that bring us a step closer to feelings of connectedness and in turn a sense of elevation. Walking, exercising, yoga or any physical activity amidst nature (outside rooms) maintaining the adequate precautionary measures of COVID-19 may again benefit the psyche, eradicating unwanted negative affect like depression and anxiety along with general sense of well-being.

The article "“Recovering With Nature”: A Review of Ecotherapy and Implications for the COVID-19 Pandemic" was retracted in 2023. Reason: compromised peer review.

Among the techniques of specific ecotherapy which focusses on interaction with wild or semi-natural areas of nature through sensory contact and mindfulness as elaborated Andy McGeeney (2), birdsong can a simple yet rejuvenating approach. Since over the recent past nature has made unique advances with social distancing decreasing the external disturbance, rare birds among other creatures have made their presence felt through their appearance. Thus, it might be an appropriate time where we might simply need to stand in solidarity and listen to birdsong savoring it. Making a birdfeeder and hanging it in our balcony, having plants that attracts insects and other butterflies, having a nature picture on the wall, some flowers in a jar by the window, buying a potted plant or growing a plant from seed can be easily done during this period of captivity. Changes in affect may be experienced on hearing the chirping of these birds and watching the non-human living beings so close amongst us. The act of bringing back to memory of a strong experience of nature, recalling that special time in nature, trying to identify what made it special, whether it is possible to find those conditions or state of mind elsewhere and if so where, can take us much away from the current distress. Observing nature as it is, finding another living plant or creature and spending time looking at it, its color, shape, texture, age, how it has adapted to its surrounding etc. without judgement would fill us with awe and a sense of wellness. Finally encouraging positive thoughts by cherishing few incidents in our lives which we are thankful for in-spite of the ongoing crisis will surely bring a sense meaning in our lives. Ecotherapy helps in conversion of loneliness to solidarity, the ability to be at peace with ourselves and our loved ones, beyond digitalization and the social noise. This has been proposed as one of the strategies to deal with the isolation and loneliness during the pandemic (143).

## Critical Evaluation of Eco-therapeutic Approach

An emerging field like ecotherapy cannot be devoid of criticisms some of which are highlighted below:

- Much more work is still left undone in terms of disorder-specific, domain-tailored systematic research as well-understanding the process through which healing occurs.
- Again all clients would not be willing to participate in such a mode of therapy due to sheer discomfort in the process or as some of the activities here may apparently appear to be ones that people are commonly engaged in.
- Finding a suitable location for many the techniques discussed above along with unfavorable weather condition may be a significant obstacle in the path of therapy.
- Use of pets or domesticated animals may be quite unsettling for some people.
- Wolsko and Hoyt (144) in their study have summarized the various obstacles in this therapeutic mode under five most frequently experienced factors that inhibited practitioners from practicing ecotherapy—lack of time and money, boundary confidentiality and legal concerns, poor location, that ecotherapy was considered to be irrelevant to treatment goals and lack of awareness and confidence in implementing ecotherapy.
- Many of these modalities are too simple to be perceived as “interventions” and hence the acceptability is ambiguous.
- The process of psychotherapeutic healing is also gradual and the socio-cognitive processes involved yet remain to be elucidated.
- Also, organized research like trials or comparative intervention studies in the field of ecotherapy poses pragmatic challenges for the lack of standardization, sampling and blinding. After all, it is nearly impossible to exclude the effects of ‘nature' on any interventions in mental health.

The article "“Recovering With Nature”: A Review of Ecotherapy and Implications for the COVID-19 Pandemic" was retracted in 2023. Reason: compromised peer review.

## Conclusion: Way Forward

To summarize, we can place our hands on the soil to feel grounded, vade in the water to feel emotionally healed, fill our lungs with fresh air to feel mentally clear, raise our faces to the heat of the sun and connect with the fire to feel the immense power within us, the sum of which is, physical connection with nature has an ameliorating effect on our mental health concerns. Indeed research so far indicates reconnecting with nature through certain unembellished methods will certainly bring about modification in the positive direction in our well-being and mental health issues.

There is some evidence to establish benefits of this therapeutic technique in various disorders (Table 1). It is important here to bear in mind that ecotherapy interventions can be simple and transformative. Dealing with the environmental crisis in the practice is of utmost importance. If we can utilize the healing properties of nature with clients appropriately it houses great potentialities for benefit. Possibilities of bringing nature into therapy rooms can be thought by the therapist as it may be a simple yet significant step (145).

In today's world where mankind's egocentric activities are resulting in environmental crisis the implication of such a therapeutic technique would be profound if it can gather momentum. Environmental and human health can be restored and considering the living world as one we can progress toward a better tomorrow. The review attempts to bring in the forefront the need of the hour which is to adopt such therapeutic techniques on a larger scale.

The article "“Recovering With Nature”: A Review of Ecotherapy and Implications for the COVID-19 Pandemic" was retracted in 2023. Reason: compromised peer review.

Considering the evidence that points out immense prospects of ecotherapy, some of its subtypes like therapeutic horticulture, animal assisted therapy, green exercise, nature art and craft and specific ecotherapy techniques involved with interaction with semi-natural areas of nature may be used to combat the psychological turmoil during this COVID-19 pandemic and the futuristic crises. This simple, pragmatic, integrative yet potentially effective psychotherapeutic technique has been neglected both in practice and research. Based on the principles of optimism, personal growth and positive psychology, ecotherapy promises a unique role in the field of social psychiatry in the days to come.

## Author Contributions

Both the authors were involved in conceptualization, literature review and drafting the manuscript. The final version was read and approved by both the authors.

## Conflict of Interest

The authors declare that the research was conducted in the absence of any commercial or financial relationships that could be construed as a potential conflict of interest.
